# The hypocretins and the reward function: what have we learned so far?

**DOI:** 10.3389/fnbeh.2013.00059

**Published:** 2013-06-13

**Authors:** Benjamin Boutrel, Nadia Steiner, Olivier Halfon

**Affiliations:** ^1^Department of Psychiatry, Center for Psychiatric Neuroscience, Lausanne University HospitalLausanne, Switzerland; ^2^Department of Psychiatry, Division of Child and Adolescent Psychiatry, Lausanne University HospitalLausanne, Switzerland

**Keywords:** hypocretins/orexins, addiction, motivation, relapse, cocaine, nicotine, alcohol drinking, opiates

## Abstract

A general consensus acknowledges that drug consumption (including alcohol, tobacco, and illicit drugs) constitutes the leading cause of preventable death worldwide. But the global burden of drug abuse extends the mortality statistics. Indeed, the comorbid long-term debilitating effects of the disease also significantly deteriorate the quality of life of individuals suffering from addiction disorders. Despite the large body of evidence delineating the cellular and molecular adaptations induced by chronic drug consumption, the brain mechanisms responsible for drug craving and relapse remain insufficiently understood, and even the most recent developments in the field have not brought significant improvement in the management of drug dependence. Though, recent preclinical evidence suggests that disrupting the hypocretin (orexin) system may serve as an anticraving medication therapy. Here, we discuss how the hypocretins, which orchestrate normal wakefulness, metabolic health and the execution of goal-oriented behaviors, may be compromised and contribute to elicit compulsive drug seeking. We propose an overview on the most recent studies demonstrating an important role for the hypocretin neuropeptide system in the regulation of drug reward and the prevention of drug relapse, and we question the relevance of disrupting the hypocretin system to alleviate symptoms of drug addiction.

## The global burden of drug addiction

“When it comes to kicking a drug habit, going through withdrawal is the easy part. The cold-turkey alcoholic shaking with delirium tremens might not agree, but only after the body detoxifies does the real challenge begin: staying clean. Ex-addicts with the strongest resolve—and plenty of external motivation in the form of frayed relationships, probationary jobs, or incipient lung cancer—struggle to resist cravings and are susceptible to relapse even years after their last dose (Helmuth, 2001).”

Quitting a drug habit is not easy to accomplish and the journey to a drug-free life is nothing but an endless personal combat to resist temptations, even long after detoxification. The inability to control drug taking is thought to be a complex disease of the brain that strikes the most vulnerable individuals and worsens with recurring drug intoxication. The use of psychoactive substances causes significant health and social problems for the people who use them, and also for their relatives. The World Health Organization (WHO) recently estimated that over one billion people were tobacco users and that alcohol disorders affected about 80 million people (WHO, 2009). In an initial estimate of factors responsible for the global burden of disease, tobacco, alcohol and illicit drugs contributed together to 12.6% of all deaths worldwide (up to 19.6% in high income countries) in the year 2000. Tobacco use and alcohol consumption are ranked the second and the eighth leading risk factors of death, respectively, responsible for 5.1 and 2.3 millions of death worldwide each year. In the U.S., illegal drug use contributes to 17,000 deaths every year, while over 400,000 people die from tobacco-related disease, and 85,000 deaths are attributable to the consequences of alcohol consumption, including alcohol-related illnesses and accidents (Mokdad et al., 2004). Illicit drug use results in the heaviest burden of mortality in the early years, whereas alcohol and tobacco use tend to take their toll much later in life, (for alcohol mostly before the age of 60, and for smoking mostly after the age of 60). Mortality statistics, however, only partially depict the picture; the frightening truth is that alcohol, tobacco and illicit drug use accounts for 19.2% of all disability-adjusted life years (DALY) in high-income countries (WHO, 2009). The DALY accounts for the burden of chronic illness on the quality of life as well as on the length of life. It thus extends the concept of potential years of life lost due to premature death to include equivalent years of “healthy” life lost by virtue of being in states of poor health or disability (WHO, 2009). In short, tobacco use and alcohol consumption were ranked the first and the second leading risk factor causes of DALYs, accountable, respectively for 13 and 8 millions of DALYs in high-income countries. Besides this unacceptable human cost, it has been recently reported that addictive disorders cost Europe €65.7 billion (Smith, 2011). It is also estimated that over 11% of US federal and state government budgets ($374 billion in 2005) are allocated to the consequences of tobacco, alcohol, and other substance use, abuse, and dependence. Finally, without alleviating their negative impact on health, it is important to note that WHO estimated that only 0.7% of the global burden of disease in 2004 was due to cocaine and opioid use, with the social cost of illicit substance use being approximatively 2% of Gross Domestic Product in those countries for which it has been measured. In brief, the treatment of drug addiction should be a priority in public health policy, and remained a challenge for both fundamental and clinical investigations.

In this context, there is a general consensus acknowledging that the reinforcing properties of drugs of abuse arise, at least in part, from a potentiation of dopaminergic neurotransmission within the mesocorticolimbic circuit. However, in the search for effective treatments alleviating signs of drug addiction, this system still is the subject of pre-clinical drug development studies but the results have been rather inconclusive or are still pending. Meanwhile, emerging data suggests that neurotransmitters other than dopamine may also play important roles in the motivational properties of drugs (Boutrel, 2008). The aim of this review is to highlight some of the recent evidence demonstrating an important role for the hypocretin (orexin) neuropeptide system in regulating the reinforcing properties of most of the categories of drugs of abuse.

## The hypocretin/orexin system in brief

The hypocretins (Hcrt, also known as orexins) are two neuropeptides, hypocretin-1/orexin-A, and hypocretin-2/orexin-B, derived from the same precursor gene produced in a few thousand neurons localized in the perifornical area (PFA) of the lateral hypothalamus (LH) (De Lecea et al., 1998; Sakurai et al., 1998). Hypocretin-containing neurons arise in the LH area and project widely in the brain with a dense innervation of anatomical sites involved in regulating arousal, motivation and stress states, where the released peptides bind to two G-coupled receptors, Hypocretin receptor 1 (Hcrtr-1) and Hcrtr-2. Their interaction with autonomic, neuroendocrine and neuroregulatory systems strongly suggests that they act as neuromodulators in a wide variety of neural circuits (Tsujino and Sakurai, 2009). In complement of a wide innervation of various neural circuits, the hypocretinergic system projects to all the major components of the extended amygdala (Schmitt et al., 2012), a brain region known to connect the basal forebrain to the classical reward systems of the LH via the medial forebrain bundle reward system. Hence, the hypocretinergic system fulfills both neuroanatomical and functional criteria to modulate critical connections that regulate both positive- and negative-reinforcing properties of drugs of abuse. However, the first compelling evidence actually established a fundamental role of the Hcrt in the regulation of arousal. Two outstanding studies unveiled the etiology of narcolepsy by linking the Hcrt system to this sleep disease using animal models (Chemelli et al., 1999; Lin et al., 1999). Further observations later established that human narcoleptic patients exhibited reduced levels of Hcrt-1 peptides in the cerebrospinal fluid and reduced numbers of Hcrt neurons (Nishino et al., 2000; Peyron et al., 2000; Thannickal et al., 2000). Nowadays, narcolepsy is still considered to be critically linked to ongoing loss of Hcrt neurons. In the current models, Hcrt stabilizes the firing of brainstem neurons that promote wakefulness and Rapid Eye Movement (REM) sleep. The Hcrt system is also thought to exert a strong and direct excitatory effect on cholinergic neurons in the basal forebrain that contributes to cortical arousal (Tsujino and Sakurai, 2009). In conclusion, the Hcrt system may be considered as a key regulator that integrates sensory inputs and orchestrates normal wakefulness and metabolic health (Sutcliffe and De Lecea, 2002; Adamantidis et al., 2007; Adamantidis and De Lecea, 2008; Schone and Burdakov, 2012). Noteworthy, a past conjecture suggested a dichotomy of reward and arousal (Harris and Aston-Jones, 2006), with a functional heterogeneity among Hcrt neurons (those in the LH regulating reward processes while those in the PFA and DMH mostly involved in the regulation of arousal and stress responses), and a functional dichotomy among Hcrt receptor signaling (Hcrtr-1 modulating reward seeking and Hcrtr-2 involved in arousal maintenance) (Gotter et al., 2012). In this regards, a recent study using functional magnetic resonance imaging reported that Hcrt receptor 1 in the striatum may specifically regulate reward seeking behaviors while Hcrt receptor 2 signaling in the cortex may preferentially modulate arousal (Gozzi et al., 2011). However, all compounds that have entered clinical development for the treatment of insomnia target both receptors, and it is important to note that, if disruption of the Hcrt transmission may cause destabilization of the boundaries between sleep states, some serious concerns may be raised regarding the use of anti-Hcrt medications for alleviating signs of drug dependence.

## Evidence for a role of the hypocretin/orexin system in drug reward

The diminished signs of precipitated opiate withdrawal displayed by Hcrt knockout mice were the first evidence linking the Hcrt system to drug addiction (Georgescu et al., 2003). This observation was confirmed a couple of years later with the demonstration that activation of LH Hcrt neurons was sufficient to reinstate an extinguished preference for an environment previously paired with morphine reward in rats (Harris et al., 2005). The involvement of the Hcrt system in the regulation of heroin intake has been recently reported (Smith and Aston-Jones, 2012), thus confirming the initial assumptions suggesting a key role for the Hcrt in mediating opiate reinforcement and withdrawal (Georgescu et al., 2003; Narita et al., 2006; Sharf et al., 2008) (see Table 1).

**Table 1:** **Summary of pre-clinical experiments demonstrating a role for Hypocretin (Hcrt) signaling in motivated behaviors**.

**Reinforcer**	**Experiment**	**Observations**	**References**
Cocaine/amphetamine	Sensitization	Chronic (but not acute) administration of SB-334867 prevents cocaine-induced behavioural sensitization	Borgland et al., 2006
		SB-334867 decreases the expression of amphetamine-induced behavioural sensitization	Quarta et al., 2010
		A dual orexin receptor antagonist (DORA-1) prevents amphetamine-induced behavioural sensitization	Winrow et al., 2010
	Self-administration	ICV administration of Hcrt-1/Orexin-A does not alter cocaine self-administration in rats	Boutrel et al., 2005; Smith et al., 2009
		Systemic and intra-VTA administration of SB-334867 reduces cocaine self-administration	Borgland et al., 2009; Espana et al., 2010
		Intra-VTA infusion of Hcrt-1/Orexin-A promotes cocaine S.A in a discrete trial and a progressive ratio schedule	Espana et al., 2011
		Systemic administration of SB334867 decreases lever pressing for cocaine reward	Hutcheson et al., 2011
		Hcrt-R1 knockout mice self-administer far less cocaine than wildtypes (WT)	Hollander et al., 2012
	Reinstatement	ICV administration of Hcrt-1/Orexin-A reinstates cocaine seeking in an operant conditioning paradigm	Boutrel et al., 2005; Wang et al., 2009
		SB334867 has no effect on established cocaine self-administration, but attenuated cocaine seeking during extinction	Zhou et al., 2012
	Conditioned Place Preference	Activation of Hcrt neuron or intra-VTA administration of Hcrt-1/Orexin-A reinstates reward seeking in a CPP paradigm	Harris et al., 2005
Ethanol	Sensitization Two bottle choice procedure	Microinjections of Hcrt-1 into the lateral hypothalamus and the paraventricular nucleus increase ethanol intake	Schneider et al., 2007
		Systemic administration of SB-334867 decreases ethanol consumption and preference in high ethanol preferring rats	Moorman and Aston-Jones, 2009
	Self-administration	Systemic administration of SB-334867 decreases ethanol self-administration in rats	Lawrence et al., 2006; Richards et al., 2008; Jupp et al., 2011a,b
	Reinstatement	Systemic administration of JNJ-10397049 (but not SB-334867) decreases ethanol self-administration in rats	Shoblock et al., 2011
		SB334867 significantly decreases yohimbine-induced reinstatement of previously extinguished ethanol seeking in rats	Richards et al., 2008
		Larger numbers of Fos-positive hypothalamic orexin neurons correlate with cues signalling ethanol availability	Dayas et al., 2008
	Conditioned Place Preference	SB-334867 reduces ethanol-stimulated activity without altering acquisition or expression of ethanol-induced CPP	Voorhees and Cunningham, 2011
		Blockade of Hcrt-2 R (JNJ-10397049) attenuates the acquisition, expression, and reinstatement of ethanol-induced CPP	Shoblock et al., 2011
Morphine/Heroin	Sensitization	Hcrt KO, WT treated with SB334867 and WT control mice display similar locomotor activity following morphine admin	Sharf et al., 2010
	Self-admin. and reinstatement	Blockade of Hcrt-1 receptors (SB334867) reduces heroin self-administration and cue-induced heroin seeking	Smith and Aston-Jones, 2012
	Conditioned place preference	Hcrt-R1 knockout mice fail to display a morphine-induced CPP, and ntra-VTA infusion of SB334867 disrupts CPP in rats	Narita et al., 2006
	Withdrawal	Hcrt-deficient mice exhibit reduced naloxone-induced precipitated signs of morphine-induced withdrawal	Georgescu et al., 2003
		Blockade of Hcrt-1 receptors (SB334867) before naloxone administration significantly attenuates withdrawal symptoms	Sharf et al., 2008
Nicotine	Self-administration	Systemic administration of SB-334867 decreases nicotine self-administration in rats	Hollander et al., 2008
		Blockade of Hcrt-1 R (SB334867) or blockade of both Hcrt-1/2 R (almorexant) both reduce nicotine self-administration	Lesage et al., 2010
	Reinstatement	Blockade of Hcrt-1 R (SB334867) (but not Hcrt-2 R with TCSOX229) decreases reinstatement of nicotine seeking in mice	Plaza-Zabala et al., 2013
	Conditioned place preference	ICV infusion of Hcrt-1 reinstates a previously extinguished nicotine-seeking behavior in mice	Plaza-Zabala et al., 2010
	Withdrawal	Somatic signs of nicotine withdrawal are attenuated in Hcrt KO and WT mice pretreated with SB334867 (but not in WT mice treated with TCSOX229)	Plaza-Zabala et al., 2012
Food/sucrose	Self-administration	SB-334867 reduces the motivation to self-administer sucrose in food-sated but not food-restricted rats	Espana et al., 2010
		Blockade of Hcrt-1 receptors (SB334867) reduces operant responding for food reinforcement	Sharf et al., 2010
		Blockade of Hcrt-1 receptors (SB334867) reduces work to self-administer high fat food pellets	Borgland et al., 2009
	Reinstatement	Blockade of Hcrt-2 receptors (JNJ-10397049) does not reduce saccharine self-administration	Shoblock et al., 2011
		ICV administration of Hcrt-1/Orexin-A reinstates food pellet seeking in an operant conditioning paradigm	Boutrel et al., 2005
		Blockade of Hcrt-1 receptors (SB334867) reduces sucrose and saccharine self-administration	Cason and Aston-Jones, 2013a,b
	Taste reactivity	Blockade of Hcrt-1 receptors (SB334867) reduces cue-induced reinstatement of sucrose and saccharine seeking	Cason and Aston-Jones, 2013a,b
		Microinjections of Hcrt-1 into the ventral pallidum hotspot enhance the hedonic impact of sucrose	Ho and Berridge, 2013
Sex	Copulatory behavior	Systemic administration of SB-334867 impairs copulatory behavior in male rats	Muschamp et al., 2007
	Conditioned place preference	Lesions of Hcrt neurons block CPP for sexual behavior in male rats	Di Sebastiano et al., 2011
Intracranial self-stimulation (ICSS) thresholds	Intracranial self-stimulation	ICV administration of Hcrt-1/Orexin-A elevates intracranial self-stimulation thresholds in rats	Boutrel et al., 2005
		Blockade of Hcrt-1 receptors (SB334867) abolishes the stimulatory effects of nicotine on brain reward circuitries in rats	Hollander et al., 2008
		Blockade of Hcrt-1 receptors (SB334867) has no effect on ICSS performance and did not attenuate cocaine effect on ICSS	Riday et al., 2012
		Blockade of Hcrt-1 receptors (SB334867) abolishes the stimulatory effects of cocaine on brain reward circuitries in rats	Hollander et al., 2012

Interestingly, Hcrt transmission also was shown to play an important role in regulating alcohol and nicotine seeking behaviors. It has been reported that the Hcrtr-1 antagonist SB334867 decreased both alcohol and nicotine self-administration behaviors in rats (Lawrence et al., 2006; Hollander et al., 2008; Richards et al., 2008; Moorman and Aston-Jones, 2009; Lesage et al., 2010; Jupp et al., 2011a,b; Voorhees and Cunningham, 2011), and that, conversely, administration of Hcrt directly into the paraventricular nucleus or in the LH increased ethanol-drinking without affecting food and water intake (Schneider et al., 2007). Strikingly, activation of Hcrt neurons also was shown to reinstate both extinguished alcohol and nicotine seeking (Hamlin et al., 2007; Dayas et al., 2008; Plaza-Zabala et al., 2013) and Hcrt signaling was claimed to trigger nicotine withdrawal as well (Plaza-Zabala et al., 2012). These preclinical observations were recently confirmed. Indeed, the Hcrt system has been involved in the affective dysregulation observed in alcohol dependent patients during alcohol withdrawal (Bayerlein et al., 2011; Von Der Goltz et al., 2011), in abstinent smokers during nicotine withdrawal (Von Der Goltz et al., 2010) and in cannabis abusers (Rotter et al., 2012).

The respective roles of Hcrtr-1 and Hcrtr-2 remain controversial though. A recent report claimed the effectiveness of the Hcrtr-2 antagonist JNJ-10397049 in reducing the reinforcing effects of ethanol, in particular in dose-dependently decreasing ethanol self-administration without affecting saccharine consumption in rats (Shoblock et al., 2011). Unexpectedly, the latter study reporting that treatment with JNJ-10397049 (10 mg/kg, sc) attenuated the acquisition, expression, and reinstatement of ethanol conditioned place preference and ethanol-induced hyperactivity in mice, also claimed that the Hcrtr-1 antagonist SB-408124 (3, 10, and 30 mg/kg, sc) did not have any effect in these procedures (Shoblock et al., 2011), whereas the studies investigating the effect of SB 334867 all converged in supporting that Hcrt-1 receptor antagonism decreases ethanol reward. A large consensus remained, however, on the role of both Hcrt receptors in preventing cue-induced reinstatement of previously extinguished alcohol-drinking behavior (Lawrence et al., 2006; Shoblock et al., 2011; Kim et al., 2012; Martin-Fardon and Weiss, 2012) (see Table 1).

With regards to cocaine, it has been established that daily pretreatment with the Hcrtr-1 antagonist SB-334867 prevented cocaine sensitization (Borgland et al., 2006) but did not block daily cocaine intake in a self-administration procedure (Smith et al., 2009). In contrast, a single injection of the Hcrtr-1 antagonist SB334867 was shown to prevent both Hcrt-, footshock-, and cue-induced reinstatement of a previously extinguished cocaine seeking behavior without however reducing cocaine consumption in a fixed ratio schedule of reinforcement (Boutrel et al., 2005; Smith et al., 2009; Wang et al., 2009; Zhou et al., 2012). Hcrt transmission may therefore selectively regulate “relapse” like behaviors in abstinent rats, but may not play any critical role in the reinforcing effects of the drug that maintain ongoing drug-taking behavior (see Table 1).

This assumption remains debatable though, since opposite observations were reported in rats trained to self-administer cocaine using a progressive ratio schedule of reinforcement, a procedure during which the number of lever presses required to earn one reward increases gradually within the session. Indeed, two studies reported that the final ratio (i.e., number of infusions) obtained by rats before termination of the session remained unchanged after infusion of the peptide or the receptor antagonist (Boutrel et al., 2005; Wang et al., 2009), whereas two other studies claimed that blockade of Hcrtr-1 with SB-334867 reduced the performance to self-administer cocaine in rats (Borgland et al., 2009; Espana et al., 2010). A striking observation, though, is that very low doses of SB-334867 (1–4 mg/kg) were shown to dose-dependently decrease cocaine self-administration in rats trained on a fixed ratio 5 schedule of reinforcement (FR5). In line with this observation, it has also been demonstrated that Hcrtr-1 antagonism dose-dependently attenuated the stimulatory effects of cocaine on brain reward systems [as measured by reversal of cocaine-induced lowering of intracranial self-stimulation (ICSS) thresholds]. Ultimately, it was established that Hcrtr-1 knockout mice (also trained on a FR5) self-administered far less cocaine than wildtype mice across the entire dose-response function (Hollander et al., 2012). Thus, a plausible explanation is that Hcrt transmission may be necessary to maintain cocaine-taking behavior when high levels of effort are required to obtain the drug, but not when the drug is readily available (Kenny, 2011).

## The hypocretin/orexin system at the interface of brain reward and brain stress pathways

Concordant observations point to a role of Hcrt-1 in driving drug seeking, in particular cocaine, through activation of the mesolimbic dopamine system. Hcrt-1 peptide has been shown to be critically involved in cocaine sensitization through the recruitment of N-Methyl-D-Aspartate (NMDA) receptors in the ventral tegmental area (VTA) (Borgland et al., 2006). Conversely, cocaine administration was recently reported to induce long-lasting, experience-dependent potentiation of glutamatergic synapses on hypocretin neurons in mice (Yeoh et al., 2012; Rao et al., 2013). Hcrt-1 peptide administered into the VTA was claimed to enhance dopamine responses to cocaine and promote cocaine self-administration (Espana et al., 2011) whereas administration of the Hcrtr-1 antagonist SB 334867 attenuated cocaine-induced enhancement of dopamine signaling (Espana et al., 2010; Calipari and Espana, 2012). Bath application of Hcrt-1 was shown to promote local dopamine release in nucleus accumbens shell slices (Patyal et al., 2012), which is in line with other reports claiming that Hcrt receptor antagonism reduced amphetamine-evoked dopamine outflow in the shell of the nucleus accumbens and decreased the expression of both cocaine and amphetamine conditioned reward and sensitization (Quarta et al., 2010; Winrow et al., 2010; Hutcheson et al., 2011).

Though, the elevated ICSS thresholds, observed after Hcrt-1 infusion into the lateral ventricle, rather suggest a decrease in excitability of brain reward systems (Boutrel et al., 2005). Indeed, such an elevation of ICSS thresholds does not match with the cocaine-induced lowering of ICSS thresholds that is considered to reflect an increased sensitivity that underlies or, at least, contributes to the positive affective state associated with drug consumption. In contrast, this long-lasting reward deficit is similar to that observed after intracerebroventricular (i.c.v) infusion of corticotropin-releasing factor (CRF) (Macey et al., 2000) or after drug withdrawal (Markou and Koob, 1991). Hence, this observation provides strong evidence suggesting that Hcrt-1 reinstates cocaine seeking by mechanisms different from increased dopamine release. In line with this observation, recent evidence suggests that intra-VTA or i.c.v administration of Hcrt-1 exerts its threshold-increasing effect via subsequent activation of the CRF system (Hata et al., 2011).

## Hypocretin and the urge for reward seeking: an allostatic adaptation in basic needs

As mentioned above, a large body of evidence demonstrates the implication of the Hcrt system in many different classes of drug reward, including cocaine, amphetamine, morphine, heroin, nicotine, and ethanol. Though, blockade of Hcrtr-1 does not evidently reduce psychostimulant consumption, whereas it quite clearly decreases both nicotine and alcohol intake in rats. Importantly, there is a consensus on the role of the Hcrt system in conditioned responding for drug-associated stimuli (context or cues), which means Hcrt may be critically implicated in addiction disease, most likely in stress- and stimulus-induced drug relapses (Boutrel and De Lecea, 2008).

However, a key question remains unanswered: how a system, that would be normally involved in the regulation of hyperaroused states in accordance with the elaboration of goal-oriented behaviors, may promote a pathological state that elicits compulsive craving and relapse to drug seeking after a period of protracted abstinence.

A recent report suggested that, in contrast to chronic calorie restriction that results in depression- and anxiety-like behaviors in rats (Jahng et al., 2007), short-term calorie restriction would promote increased arousal, increased locomotor activity and decreased anxiety-like behaviors that could be attributed to the activation of the Hcrt system. This antidepressant-like response would be lost after chronic calorie restriction due to a downregulated expression of prepro-Hcrt mRNA in the LH (Lutter et al., 2008). Thus, in healthy physiological conditions, the Hcrt system may contribute to a resilient-like state by reducing depression-like symptoms induced by short-term calorie restriction, whereas a compromised Hcrt system upon chronic calorie restriction may contribute to worsen signs of anxiety and depression (Rotter et al., 2011). Our idea is that a similar adaptation may occur during chronic drug consumption (and the concomitant recurring drug withdrawals). Indeed, it is well accepted that Hcrt elicits appropriate levels of alertness to engage exploratory behaviors and strengthen motivation for food seeking depending on physiological needs (hunger, thirst). Similarly, at cessation of drug consumption, the Hcrt system may act as an alarm signal that would prepare the organism for withdrawal and face the consequences on energy and fluid homoeostasis (such as starvation activating the Hcrt and eliciting food seeking to prevent caloric restriction). This assumption is in line with the diminished signs of precipitated opiate withdrawal displayed by both mutant mice deficient in Hcrt (Georgescu et al., 2003) and C57BL/6J mice treated with a Hcrtr-1 antagonist (Sharf et al., 2008). We thus consider that chronic drug intoxication may induce changes in basic needs priorities, and that the Hcrt may contribute (as a means to maintain stability of the internal milieu in case of dependence) to a particularly vulnerable state of the brain that may trigger the urge for drug seeking and drug taking, even long after last consumption and withdrawal (Boutrel et al., 2010). A new role would be assigned to the Hcrt system, no longer for fine tuning arousal and goal-directed behaviors in response to metabolic needs, but for eliciting the hyperaroused and motivated state, if not anxious-like state (Plaza-Zabala et al., 2010), required for optimizing drug seeking, in other words drug craving (Martin-Fardon and Boutrel, 2012).

Since Hcrt fibers have been shown to innervate both the NAcc (Baldo et al., 2003) and the insula (Hollander et al., 2008), it is tempting to speculate that Hcrt may contribute to define behavioral strategies by optimizing the processing of environmental signals in attention-demanding tasks with regard to past experiences. Hence, the Hcrt system may enhance cognitive arousal and attention for improving prediction making, and drive sustained attention for achieving the goal-oriented behavior whatever the context is: reward seeking or punishment avoidance (Berridge et al., 2010). In line with this interpretation, a recent study established that cues previously paired with cocaine consumption elicited a significant increase in cFos-positive Hcrt neurons compared to cues previously paired with sweetened condensed milk. Further, following the extinction, the number of Fos-positive Hcrt cells was decreased in cocaine rats compared to drug naïve ones and those exposed to the sweetened condensed milk, suggesting a decreased activity in Hcrt neurons of rats with a history of drug abuse. Strikingly, the Hcrtr-1 antagonist SB334867 was shown to reduce cue-induced cocaine seeking at lower doses (starting at 3 mg/kg) than those used for preventing cue-induced sweetened condensed milk seeking (Martin-Fardon et al., 2010). Again, chronic drug intoxication may induce changes in basic needs priorities, and the Hcrt system may be part of a common mechanism for adapting and/or ranking priorities and eliciting appropriate levels of alertness to drive attention processes and trigger goal-directed behaviors according to these new priorities.

## Potential consequences of a pharmacological disruption of Hcrt transmission

With the accumulation of preclinical evidence demonstrating a role for Hcrt in the maintenance of arousal, several pharmaceutical companies have developed Hcrt receptor antagonists for the treatment of insomnia. SB-334867 was the first Hcrtr-1 antagonist developed by GlaxoSmithKline (GSK) in the late nineties and remains to date the most studied Hcrtr-1 antagonist. Several other Hcrtr-1 and Hcrtr-2 antagonists, consensually called SORA for Single Orexin Receptor Antagonists, as well as ligands with similar affinity for both receptors, also called DORA for Dual Orexin Receptor Antagonists, have been developed then. Exhaustive reviews covering patent literature published between 1999 and 2009 have been recently issued (Coleman and Renger, 2010; Scammell and Winrow, 2011). But these technical reports focused mainly on the chemical properties of these compounds. Further therapeutic opportunities offered by Hcrt ligands have been recently examined, however these reviews of the literature cover essentially the pharmacology of sleep and arousal (Coleman and Renger, 2010; Scammell and Winrow, 2011). Very few compounds have entered clinical development. Actelion, in partnership with GSK, has been conducting Phase III studies with the DORA almorexant for the treatment of insomnia, and Merck reported that the DORA MK-4305 (Suvorexant) entered into Phase III development for treating insomnia and claimed encouraging preliminary studies with the DORA MK-6096 (DORA-22) (Coleman et al., 2012; Herring et al., 2012; Willyard, 2012; Mignot, 2013; Sun et al., 2013; Uslaner et al., 2013). Nevertheless, it has not been yet reported any clinical investigations with one of these compounds for treating drug addiction. Thus far, little is known on the putative adverse effects of Hcrt receptor antagonists. Nevertheless, a rapid review of the available evidence allows us to raise a few concerns about the effects of a pharmacological disruption of the Hcrt transmission (Scammell and Winrow, 2011).

In addition to the prominent role of the Hcrt system in arousal stability, Hcrt have been suggested to play a key role in driving arousal and goal-oriented behaviors (Boutrel et al., 2010). Briefly, compelling evidence has established a role for the Hcrt in enhancing cortical arousal and attention, particularly with regard to limbic and visceral states (Huang et al., 2006). In particular, Hcrt cells were shown to discharge with maximal activity during exploratory behavior, which can be considered as sustained attention or alertness (Mileykovskiy et al., 2005). Confirming this idea, systemic or intracerebral administration of the Hcrtr-1 antagonist SB 334867 has been shown to disrupt attention in rats (Boschen et al., 2009). In line with these preclinical reports, recent clinical observation reported that narcoleptic patients exhibited attention deficits that cannot be attributed to sleepiness only (Rieger et al., 2003). Disruption of Hcrt signaling might therefore constitute a risk for developing attention deficits and quite serious long-term debilitating effects.

Further, Hcrt neurons are sensitive to glucose, leptin, triglycerides, and carbon dioxide concentrations, and have long been considered to maintain physiological levels of caloric intake. Nevertheless, recent evidence suggests that Hcrt do not seem to be critical players in food intake behaviors, but rather adapt arousal and motivation levels to allow feeding and drinking behaviors (Tsujino and Sakurai, 2009). Depending on physiological needs (hunger, thirst), Hcrt elicits appropriate level of arousal to engage exploratory and goal-oriented behaviors. This can ultimately strengthen motivation for palatable food and liquids (Kunii et al., 1999; Thorpe et al., 2005; Borgland et al., 2009) or lead to the reinstatement of a previously extinguished food seeking behavior in an operant conditioning paradigm (Boutrel et al., 2005; Nair et al., 2008). Consistent with this possibility, the inhibitory effects of SB-334867 on consumption of a palatable reinforcer (high-fat chocolate food) were recently suggested to be dependent upon the level of effort necessary to obtain the reinforcer (Borgland et al., 2009). Indeed, intra-LH Hcrt-1 had the greatest effects at higher effort-requiring schedules, whereas Hcrtr-1 signaling appeared to have little involvement in responding for high fat or sucrose pellets in low effort situations (Thorpe et al., 2005; Borgland et al., 2009). Nonetheless, recent findings using a pharmacological disruption of Hcrt transmission have shown that Hcrtr-1 plays an important role in the motivation to respond for both food (Sharf et al., 2010) and sweetened taste (Cason and Aston-Jones, 2013a,b), confirming that Hcrt neurotransmission is as critical for modulating the reinforcing and conditioned rewarding effects of non-drug reinforcers as it is for drugs of abuse. Thus, disrupting the Hcrt system may represent serious concerns with regards to appetite regulation.

Besides, it seems that the Hcrt do not drive alertness elicited by physiological needs only, but in response to psychological needs as well. Indeed, concordant evidence has recently suggested that Hcrt may potentiate male sexual behavior in rats (Gulia et al., 2003; Muschamp et al., 2007; Bai et al., 2009; Di Sebastiano et al., 2010, 2011; Di Sebastiano and Coolen, 2012) in a way that facilitates the energized pursuit of sexual engagement. Strikingly, higher Hcrt-1 content was found in mid brain, medulla and thalamus harvested at late proestrus relative to all other stages of the sex cycle in female rats (Russell et al., 2001). These observations are considered to reflect greater release of Hcrt-1 into nerve endings in brain areas implicated in sex cycle-specific behaviors, such as lordosis and sexual receptivity in female rats (Russell et al., 2001). Therefore, Hcrt may promote sexual arousal in both male and female rats. Interestingly, the main reinforcing behavior in females is considered to be maternal care. Not surprisingly, Hcrt-1 modulates maternal behavior in mice (D'Anna and Gammie, 2006). Hence, not only does Hcrt drive appropriate levels of alertness in response to thirst and hunger, but also it triggers sexual arousal and sustained maternal care. It is then tempting to suggest a role for Hcrt in adapting/strengthening coping strategies in animals facing desire and needs. Again, this observation may raise quite a few concerns with regards to a long-term disruption of the Hcrt system.

## Conclusion

The Hcrt system controls sleep and wakefulness through multiple interactions with brain structures involved in the regulation of emotion, reward, stress, and energy homeostasis. A consensus has emerged on the role of Hcrt in eliciting appropriate levels of arousal to engage exploratory and goal-oriented behaviors depending on physiological needs. Our hypothesis is that chronic drug intoxication may compromise these basic needs priorities, and the Hcrt system may become “hijacked” and consequently, may drive drug-oriented behaviors according to these new priorities. This assumption is supported by a large body of evidence demonstrating a role for the Hcrt system in drug reward, particularly in “relapse-like” behaviors in abstinent rats. Further, converging data now suggest a role for Hcrt in the affective dysregulation observed in dependent patients during alcohol and nicotine withdrawal. Still, it remains unclear whether Hcrt antagonism may offer a clinical opportunity for reducing alcohol and nicotine (and possibly opiate) consumption in dependent patients. Unfortunately, it appears quite clear that disrupting the Hcrt system most likely will not reduce cocaine or amphetamine intake. A large consensus remains though on the possibility to treat dependent patients with Hcrt receptor blockers for alleviating symptoms of drug dependence, notably the urge for drug seeking during protracted abstinence from most major drugs of abuse. As reviewed above, the beneficial effects of such a medication may be limited by some serious side effects among which sleepiness, decreased appetite, attention deficits, and reduced libido. In conclusion, there is considerable evidence that the Hcrt system is key to many aspects of reward seeking behaviors and, thus, could be a useful target for controlling relapse for drugs of abuse. However, the fundamental role of these systems in more basic aspects of homeostasis and non-drug reinforcement need to be carefully considered in order to ensure that unintentional adverse consequences are not presented.

### Conflict of interest statement

The authors declare that the research was conducted in the absence of any commercial or financial relationships that could be construed as a potential conflict of interest.
